This article has been retracted.

# Detection of WBC, RBC, and Platelets in Blood Samples Using Deep Learning

**DOI:** 10.1155/2022/1499546

**Published:** 2022-07-14

**Authors:** Lamia Alhazmi

**Affiliations:** Department of Management Information System, College of Business Administration, Taif University, P.O Box 11099, Taif 21944, Saudi Arabia

## Abstract

A blood count is one of the most important diagnostic tools in medicine and one of the most common procedures. It can reveal important changes in the body and is commonly used as the first stage in the process of evaluating patients' health. Even though this is a common practice, delivering examinations in laboratories can be difficult due to the availability of expensive technology that requires frequent maintenance. This study is developing an alternative deep learning computational model capable of automatically detecting cells in images of blood samples. Using object detection libraries, it was possible to train a model that was focused on this task and capable of detecting cells in images with adequate accuracy. When the identification of cells in images of blood samples was taken into account in the best results obtained, it was possible to count white cells with an accuracy of one hundred percent, red cells with an accuracy of 89%, and platelets with an accuracy of 96%, which generated subsidies to develop the primary components of a blood count. The components that were supposed to classify the various types of white cells were not carried out due to the limits of the dataset provided. On the other hand, the study can be broadened to include further works that deal with this issue because it produced satisfactory results.

## 1. Introduction

Health is an important pillar of society, and assisting others is becoming increasingly important. Given the challenges and conditions of the COVID-19 outbreak, it is vital to automate procedures to speed up health professionals' work and focus on emergency care. Automation has grown increasingly important in numerous industries as technology and communication have advanced. Because of the epidemic, laboratory testing has increased, necessitating more health experts' attendance, analysis, and reporting [1, 2]. There is an overflow of functions because not every location has adequate workers to manage this. This research tries to detect blood images to aid in the creation of blood counts, creating a tool for health-care providers. Blood counts are performed using pricey, specialized equipment. To automate this procedure, deep learning algorithms can replace specialized equipment.

Deep learning (DL) algorithms are employed in various fields, including medical, economics, education, e-commerce, and virtual games. DL is emerging as a viable alternative to traditional job execution and automation methods [3, 4]. Deep learning is being used in some health-related projects to improve decision-making. Deep learning makes use of enormous amounts of data. This data must be collected and preprocessed for deep learning to be effective. The deep learning model is trained and tested with other data to produce results, then postprocessed for better visualization, and delivered to the health professional.

This article analyzes blood test photos to detect and count cells automatically. Because the method is manual, these samples are checked and analyzed using glass slides and a microscope to establish blood counts. Larger labs also employ costly counting machines. This research utilizes a huge collection of images of blood samples to recognize and to count the many types of cells in the sample, assisting clinicians in preparing blood counts. Given the variety of deep learning algorithms and their uses, how could a computational model for detecting and counting cells in blood sample photos assist laboratory and health-care professionals?

## 2. Theoretical Approach

### 2.1. Artificial Intelligence: Machine Learning and Deep Learning

The deep learning technique, which is the focus of this study, is one of the subfields of machine learning, which is itself a subfield of AI. As a result, the concept of artificial intelligence must be taught before digging into each of these concepts, their differences, and applications. Artificial intelligence is a means of solving issues of many types in an automated manner, that is, without the assistance of a human or a specific user. People are seeking novel ways to automate routine tasks; therefore, this sector is garnering a lot of attention these days [5, 6]. This method is used in a variety of businesses and is now being applied in homes for a variety of reasons. This research aims to figure out how to teach machines and computers to have intelligence that is becoming more human-like. This is usually performed using pattern recognition, which allows computers to be trained to analyze and understand data in a way that is comparable to how people learn. On the other hand, machines usually need a lot of data to understand something simple.

#### 2.1.1. Machine Learning

Problem resolution using computational tools and methods designed for specific goals is common, but not in all circumstances because a single line of steps is not always known. To be resolved, a machine learning model can forecast when the data input and the desired result are known, but not the means to get there. We know the parameters and method for obtaining the result in traditional programming methods, but with machine learning, the machine learns and presents the approach (ETHEM, 2016) [7]. Every machine learning model goes through data preparation, training, and testing. Preprocessing is the examination and modification of data in order to improve model comprehension by removing extraneous information and changing the format (RASCHKA, 2015). Before forecasting any value or outcome, the machine learning model must be trained using the specified approach. The person in charge of training must provide a substantial amount of data and the expected results in each, as well as the training parameters and settings. As a result, the model learns to understand and interpret data, and it can predict future data outcomes (RASCHKA, 2015).

The testing follows the model training. The accuracy, precision, and recall of the model are measured in this step. The accuracy of the model reveals how many classes it correctly classified. Precision indicates how many correct positive classifications there are. The recall metric indicates how many positive expected value classifications are correct. The F1-score is a summing of precision and recall (NICK, 2018).

A confusion matrix describes the number of hits and errors associated with true or false positives and true or false negatives for easy display and calculation.

*(1) Traditional Algorithms*. There are two types of machine learning techniques: supervised and unsupervised. In supervised learning, the correct result or where the model should originate from the data is known; however, in unsupervised learning, the model must deal with unstructured input and no obvious outcome (RASCHKA, 2015) [8].

Both regression and classification are supervised learning techniques. Regression methods forecast actual values, whereas classification models categorize data (RASCHKA, 2015).

Methodologies for data regression may be listed (NICK, 2018).

- Linear regression is a simple and traditional method for predicting regression involving drawing a line through the data. Multiple linear regression employs additional variables, whereas polynomial linear regression employs variables with exponentiation to produce a more aggressive outcome
- Decision tree: This strategy uses model-learned criteria to forecast values. To find patterns in the known data, divide it into related groups

Random forest combines the processing capacity of numerous decision trees to get a more thorough and accurate result.

A list of data classification algorithms is available (RASCHKA, 2015).

- K-nearest neighbors (KNN): This algorithm classifies data by comparing it to similar data. It is lazy since it does not present an intelligent model; it just saves and compares facts
- Decision tree classifier: Decision trees, like regression, predict classes for specific data based on learned criteria. These criteria will be taught by grouping known data into similar groups in order to find patterns, which in this case, are the necessary classes for interpretation
- Random forest classifier: Random forest, like regression, combines the processing capabilities of many categorizations decision trees to produce more accurate output

A nontraditional approach, neural networks, can be used for regression and classification. This project will investigate an alternative to standard algorithms.

*(2) Neural Networks*. Neural networks use perceptrons, a computerized representation of a neuron, to mimic the human brain. The perceptron can receive inputs (data) and output. Using numerous perceptrons in a network improves their performance by combining their processing power and achieving a faster, more accurate output. An artificial neural network (ANN) is this structure.  Figure 1 shows the structure of a perceptron, where *x*  is the input, *w* is the weights, *Σ*  is the sum, *f* is the activation function, and *y* is the output [9]. An artificial neural network (ANN) is a structure built using perceptrons to mimic human brain processing. Its structure is defined at several levels, with an input layer, an output layer, and hidden intermediary layers responsible for overall processing, each with a programmable number of perceptrons.  Figure 2 depicts this structure, which includes input, hidden, and output layers. The selected weights are as important as the information transmitted from perceptron to perceptron. Weights are defined values for each piece of information received by the perceptron and are changed to produce the desired output. An ANN can learn to do a variety of tasks, such as classification, by employing a backpropagation strategy that adjusts the model's learning rate in phases.

First, the algorithm uses random weights to train the artificial neural network. During training, the algorithm predicts outcomes that are then compared to the correct numbers to determine success. The backpropagation algorithm calculates the difference between the result and the true result and feeds this error information to all preceding layers in order to alter weights and reduce error [10]. This process is done several times during training until the changes induce an increase in inaccuracy, indicating that the weights have reached their maximum. This stage of modifying the weights of the network is critical because it helps the model learn from its failures.

### 2.2. Deep Learning

In some cases, machine learning is insufficient for data learning because learning occurs through pattern recognition based on data that cannot be used in any case, must be prepared and adapted for each model, or the machine cannot learn on its own because it always requires human intervention to process the data. Deep learning is required to emulate human reasoning. Deep learning uses deep neural networks to enhance neural networks (DNNs). Deep neural networks (DNNs) are deep learning neural network architecture with more neurons, hidden layers in more intricate topologies, and specific neuron connections [11]. Deep neural networks created intriguing versions that focused on a certain specialism, emulating human nature in order to accomplish tasks and produce intelligence. Some of these types are related to natural language processing, such as RNNs, or image recognition and interpretation, such as CNNs.

#### 2.2.1. Recurrent Neural Networks (RNNs)

Recurrent neural networks are a type of neural network designed to evaluate temporal input sequentially. They can forecast variables in relation to time. Its topology facilitates feedback connections of passed-on information; loops allow the information to remain as if the network were repeated. RNNs make use of information in a predefined sequence, such as updated data.

#### 2.2.2. Convolutional Neural Networks (CNNs)

Convolutional neural networks are a type of neural network architecture created for image recognition that can break down images and analyze them. This network represents height, width, and color as three-dimensional matrices.

Traditional DNNs work well for small images, but with a large amount of data, each pixel in the image, the model would struggle to learn; hence, CNNs were developed. CNNs were constructed with partially connected layers and significant weight reuse to address this issue, resulting in fewer parameters to understand and pass on faster training and less training data required [12–14]. This efficiency is also due to the fact that, unlike DNNs, when a CNN learns to interpret an image feature, it can identify that feature wherever in the image. DNNs are more specialized than CNNs.  Figure 3 depicts the convolutional layer at the start of the procedure.

#### 2.2.3. Libraries and Resources

Some market-available free libraries assist with deep learning's essential architectures and resources. Tensorflow and Keras are Python and C++ libraries that can communicate with one another and are widely used in the deep learning field (GIANCARLO; REZAUL, 2018).

Tensorflow is a machine learning platform that is open source and focuses on neural networks and deep learning. Keras is the foundation for Tensorflow's neural network APIs. In 2018, Google's Keras library was included in Tensorflow (2021, TENSORFLOW).

Keras focuses on deep neural networks for rapid prototyping and testing. It is straightforward, modular, and extendable. It has layers, loss functions, activation functions, and other features. It also has convolutional and recurrent neural network modules (KERAS, 2021).

The combination of two machine learning and deep learning libraries creates an extremely beneficial tool for this objective, allowing users to work with numbers, text, audio, and image data [15, 16].

Tensorflow documentation can help you learn how to build a convolutional neural network, providing theory and a practical example. The documentation for this package enables image classification based on a dataset (TENSORFLOW, 2021).

You can also work with different library modules in Tensorflow; object detection was utilized here. This module is responsible for detecting picture objects. Instead of detecting everyday objects, the model is trained to recognize and to differentiate between cells in a picture.

Object detection facilitates image processing and computational model processing while also providing useful training tools. Tensorflow's object detection module was used throughout the model training phase.

## 3. Material and Methods

### 3.1. Dataset

Choosing the dataset for AI work is critical because it influences all subsequent methods. During the search, the best contender for the dataset was the BCCD Dataset (SHENGGAN, 2019).

This dataset was chosen since it is cited in numerous papers. This is the most comprehensive and in-depth dataset for this research area according to the literature. Another important factor was the availability of high-quality pictures for visual interpretation and training deep learning models. WBC (white blood cell), RBC (red blood cell), and platelets are included in the dataset. All of the photos are in one folder, and the XML coordinates for each cell are in another. The investigation into its resources and limits began with the dataset in hand. One of the dataset's limitations is that not all picture cells have mapped coordinates. The dataset contains cells with no coordinates, which can make model training difficult [14].

White cell classification is missing from this dataset. In photos, the dataset distinguishes white, red, and platelet cells. This is insufficient for a complete blood count. In order to provide a more accurate patient diagnosis, white blood cells must be classified (neutrophils, basophils, eosinophils, lymphocytes, and monocytes). White cell classification could be future research.

After getting the dataset, images were modified for model detection. The repository includes images as well as Python data processing programs to demonstrate the dataset's utility. A program outlines cells for a data preview. Because this effort contains deep learning, the data processing will adhere to its specifications. All Python files in the dataset were eliminated, leaving only the images directory and the XML files directory with image coordinates.

### 3.2. Object Detection

The computational model's resources were trained and configured using Tensorflow. Tensorflow contains a large number of functions and utilities for machine learning and deep learning, so selecting the proper ones is critical. Object detection is one of the most exciting components for this job (TENSORFLOW, 2021).

Tensorflow's object detection module locates previously learned picture portions. It recognizes people and things in photographs. It can also be used to recognize people, vehicles, animals, and other common components in security cameras in films, frame by frame. This project develops a computer vision system that can detect cells in a photograph, count them, and generate a hemogram [17]. This is where the object detection module comes in. This module is typically used to detect people and things, but it can be customized to learn about blood contents. When the model is trained on a large number of blood images, it may learn from the data and make predictions.

Understanding the library's resources and limitations required extensive documentation. The object identification module had less documentation, but it was useful for a variety of project issues, particularly base codes. The first codes were written using the test cases from the documentation, which provided a solid introduction of the computational model's numerous setups and general behavior.

An environment must be established in order to optimize code execution. The algorithm must be configured to run on the GPU rather than the CPU, which is the default. GPUs provide superior image processing results in less time, especially in large quantities.

The environment was prepared by installing CUDA. The NVIDIA CUDA platform uses parallel computing to optimize graphics card processing and speeds up applications. Use cuDNN in addition to CUDA. cuDNN is a deep neural network library that enables the use of neural network design with machine learning methods, making it appropriate for this job. CUDA improves the efficiency and quality of cuDNN (CUDA, 2021; CUDNN, 2021).

The algorithm can be executed once the environment is ready. At this stage, the documentation's basic examples were run to see how the algorithm behaved on the system, the sample processing outputs, and how long they would take. This step was critical for the project's continuation because it allowed for better planning of the next stages.

### 3.3. Computational Model

The dataset was placed into the model's training and image recognition templates after the resources, libraries, and environment were in place. The photographs were large enough for the algorithm and had the same size and magnification scale. Import and translate XML files into model-readable variables before recognizing image coordinates. The data in the files and the data accepted by the model were of varying scales and proportions. The algorithm was unable to locate the picture cells during import. A function to translate XML coordinates into model scale numbers was required to adopt this method, allowing coordinates and images to be loaded [18].

Thus, a key test for one cell type initially produced satisfactory results with low success rates without modifying the model features. To maximize model notions, the following qualities had to be changed:

- Batch size: The size of the training batch. Larger batches enhance learning but necessitate more machine processing
- Learning rate: The learning rate of the model. Larger groups learn more quickly. If it becomes too large, the model begins to recognize bogus cells. The model cannot find cells if it is too small
- Batches: The number of algorithms passes (also known as epochs). The training interval of the algorithm is defined here
- Hit percentage: A hit occurs when the algorithm is more than 50% certain about a cell

To configure these parameters, each code execution was tested and tweaked. This was repeated until the best values were discovered.

This job necessitates the selection of a pretrained neural network in addition to establishing these settings. Training new models is sped up by leveraging a pretrained network. If it were properly trained with simple information like outlines and common features, the results with more intricate aspects would be better.

This experiment uses the “resnet50” network, but the object identification module accepts a variety of others. This decision was influenced by image size and network speed tests (HE et al., 2015).

“resnet50” aids in the training phase of the model because just the last layers must be learned. Because the model's early layers were already trained with generalities, only the last levels require specific data. After teaching one type of cell, train the others with blood sample photos. First, all cells were trained simultaneously, which took too long and yielded poor results.

This necessitated a different approach. Instead of training all cells at once, a model for white cells, red cells, and platelets was created. This made training more efficient and specific to each type.

Because three models are used, inputting an image for verification in predicting results will result in three separate responses, one for each cell type. This technique allowed for different parameter values for each class, enhancing results. Because this project aims to count individual cells, splitting the models for each cell has no effect on the final result.

### 3.4. Evaluation

Metrics were used to assess the computational model's performance and the output of each trained model. To compare choices, each model option used various metrics and parameters. As a result, it was feasible to determine the best algorithm for the prototype and the best settings to maximize its performance. The first evaluation metric was test accuracy. They were also measured using MSE and rMSE (mean squared error). rMSE (root mean squared error) is an MSE variant that employs the square root. First, the standard accuracy was determined by comparing the number of real cells expected to be discovered by the model to the number discovered. Based on these values, the ultimate accuracy percentage was computed. The MSE formula is shown below. Finally, the mean square error is calculated by averaging all the data.

(1) $$\begin{array}{c} \text{MSE}=\frac{1}{n}\overset{n}{\underset{\underset{\text{Test set}}{\underset{⏟}{i=1}}}{\sum }}{\left(\underset{\begin{array}{c} \text{Predicted}\\ \text{ Value} \end{array}}{\underset{⏟}{y_{i}}}-\underset{\begin{array}{c} \text{Actual }\\ \text{Value} \end{array}}{\underset{⏟}{{\overset{\wedge }{y}}_{i}}}\right)}^{2}. \end{array}$$

The ideal value of this number is close to 0, as the higher the number, the greater the model error. As a result is always squared, predictions far from the real are easily noticeable, making this metric interesting for problems where large errors are not tolerated. The rMSE was calculated based on the formula presented below. As the MSE was already calculated, it was possible to calculate the resulting square root to find the final rMSE.

(2) $$\begin{array}{c} \text{rMSE}=\sqrt{\frac{1}{n}\overset{n}{\underset{\underset{\text{Test set}}{\underset{⏟}{i=1}}}{\sum }}{\left(\underset{\begin{array}{c} \text{Predicted}\\ \text{ Value} \end{array}}{\underset{⏟}{y_{i}}}-\underset{\begin{array}{c} \text{Actual }\\ \text{Value} \end{array}}{\underset{⏟}{{\overset{\wedge }{y}}_{i}}}\right)}^{2}}. \end{array}$$

This metric is a complement to the normal MSE, because, through this metric, it is possible to measure the final result without changing the scale of the error, facilitating some comparisons. For a while the MSE is squared, the rMSE does not have this problem, as the square root is extracted in the final process.

### 3.5. Prototype

Following the definition of the best viable instance of the computational model, it was exported and used to create a working prototype. The Tensorflow library documentation was examined to understand checkpoints before exporting the model. Checkpoints in Tensorflow save the state of a trained model for later use. As a result, a ready-made model can be employed without retraining for picture predictions only. To use the model elsewhere, simply import a file. The AI algorithm prototype was created using Streamlit. The Streamlit framework in Python makes prototyping simple and quick. A web app with few commands allows you to concentrate on development. As a result, the graphical user interface is unimportant. It is simple to customize, displaying all of the algorithm's capabilities on the screen and allowing the user to give input data and see the algorithm's output (output). This enables user engagement in real time.  Figure 4 depicts the interface of the prototype.

The user can send a link to an Internet image in the format of the dataset where the model was trained, as seen in the prototype. The recognition of white, red, and platelet cells in a blood sample using the trained model is illustrated in Figure 4. Additionally, aggression percentages for each cell detection can be calculated.

## 4. Results and Discussion

### 4.1. Model Performance Analysis

The dataset used as a basis for this work has 364 different images of blood samples. Each image can contain up to 30 cells of different classes located in different image portions. The classes used in this research are red cells (RBC), white cells (WBC), and also platelets (platelets), which are identified through coordinates that indicate the location of each cell in the image and are stored in XML files that accompany the dataset in question.

This dataset was separated into two main groups. The first group refers to the set of images aimed only at training, with 80% of the total images; this group contains 291 randomly selected images, while the second group aimed only at testing, with 20% of the total images, which contains 73 separate images for this purpose. As the training group needs to be larger to have good training of the model and finally to test the remaining images, the selection of 80/20 of the separation of the files was adopted. The model was configured following a few key principles and configurations. First, the pretrained neural network with the best result and performance for this image group was selected, “resnet50”, recognized in the code base by “ssd_resnet50_v1_fpn_640x640_coco17_tpu-8.” In addition to this choice, four fundamental parameters were carefully selected, seeking the best performance in the shortest time. The definition of batch size, learning rate, number of batches, and the percentage of base hit can be seen in Figure 5.

After model training, predictions were measured using 3 different metrics. The first was standard accuracy, which allows for an overview of the progress of the process. Carrying out the standard accuracy measurement, considering the number of real cells and the number of cells that should be found by the model, the following relationship was arrived at, using the best possible result as a parameter:

- WBC: 74 cells found from 74 real cells (100.00% hit and 0.00% fail)
- RBC: 1,007 cells found from 908 real cells (89.10% hit and 10.90% fail)
- Platelets: 57 cells found from 59 real cells (96.61% hit and 3.39% fail)

The MSE and the rMSE are complementary metrics that are easy to use and refer to the performance of the computational model. While the MSE works by calculating the mean square error, the rMSE is the root of this value found. Such metrics are interesting because they allow you to visualize considerably, even small errors. This scale does not have a maximum or ideal number, but the result should approach zero; the closer, the better. Thus, using the formulas from the previous sections, it was possible to arrive at the relationship in Figure 6. Through the relationship in Figure 6, it was possible to perceive that the best performance is in the detection of white cells, which is in line with the definitions found by the accuracy seen above. This may have happened because, in the dataset, in most of the images, there is at least one white cell that is easily detected about the others. Following this, platelets also show good results, similar to the model's accuracy relationship. Finally, the red cells present inferior results about the others. This may have happened because of their abundance in all images, while the other classes have one or two cells per image, the red cells may appear in a number greater than 20, which makes it difficult to learn the model and hinders the prediction in this case.

### 4.2. Identification of White Cells (WBC)

The first class of cells worked from the first test using the dataset were white cells. This was due to its easy identification about the others, being a great candidate to start the tests and later the first versions of the prototype.

These cells are present in the images in low quantity, as the dataset sought to focus on a white cell in each image. Although it is possible to find even two or three in some cases, in addition to the quantity, they can be distinguished from the others through their coloring.

In Figure 7(a), the model's detection of the white cell can be observed where it was possible to differentiate and delimit the cell satisfactorily. In Figure 7(b), the same process can also be observed, but in a different situation.

It could be seen that the model had a good hit rate, taking into account both performance metrics and visual analysis of the images. In this way, it is possible to perform cell counts with a good assertiveness index.

### 4.3. Identification of Red Cells (RBC)

After the detection of white cells, the next step was the interpretation of red cells. These differ in their detection in relation to the others due to their quantity. Red cells appear in a greater proportion, with more than 20 cells per image.

A large amount of these types of cells is a challenge for the model, mainly due to the delimitation of their areas. As they do not have a defined shape and often overlap, this hinders their identification.

In Figure 7(c), we can visualize the detection process of red cells. It is possible to count the cells as necessary, with a small margin of error.

However, in Figure 7(d), it is also possible to visualize the identification by the model. However, even with the overlapping of cells at a higher density, the model still managed to identify most of the cells correctly.

It is possible to conclude that although it does not have as positive performance as the other classes, the results are also good as they allow a red cell count with a small margin of error.

### 4.4. Identification of Platelets (Platelets)

Finally, platelet detection was performed in a similar way to white cells. Despite being more present in the dataset than the white cells, they are not as high in number as the red cells, presenting small sets by images. Another characteristic factor about the others is its size, which is much smaller and easy to identify with the naked eye.

Although they are easily identified, overlapping cells can also happen in this case, hindering the performance of identification by the model. But this happens in a significantly smaller number compared to red blood cells.

It is possible to visualize in Figure 7(e) the process of identification of platelets, where the model presents a performance considered great.

Figure 7(f) shows a slightly different situation. In this analysis, the model was able to identify the 4 platelets that appear in the image correctly, but with a slightly reduced assertiveness margin of the algorithm.

With this, we can conclude that platelets have adequate performance in their identification, allowing a satisfactory count. Although not as positive as in the detection of white cells, it still outperforms red cells in terms of performance and assertiveness criteria.

### 4.5. Elaboration of Hemogram Elements

It is feasible to generate elements of the hemogram based on the identification and counting of cells, as seen above. A blood count is essentially a count of cells followed by comparing the results to precalculated indices of optimal values for each patient type.

After identifying the cells, the initial values of the blood count can be calculated by counting each kind. The units of measurement are critical in this process since they differ for each type of cell. The cubic millimeter (mmS), a unit of volume, serves as the foundation for the calculation. The count is performed in proportion to one cubic millimeter to compute the leukocytes, which are white cells, and the platelets. However, because erythrocytes, or red blood cells, are in higher abundance than other cells, the computation of millions of cells in a cubic millimeter is conducted.

The erythrogram can be created by multiplying the erythrocytes by millions/mmS. The number of leukocytes found in unit/mmS can be used to create the leukogram. Finally, a platelet count based on the number of platelets recognized in units/mmS can be calculated.

This data is required to diagnose various disorders and abnormalities in the patient's body. For example, the leukogram is the primary test used to assess a person's immunity by measuring the number of leukocytes present in the body. Platelet count also reveals a lot about the body, measuring the individual's blood clotting and bleeding proclivities. In addition to the low amount of red blood cells, it could suggest anemia or another condition, among many other possibilities.

We may conclude that with this data, we can create significant aspects of the hemogram that, when applied to a sample with volume values, will be useful and fascinating to use. When the values provide different outcomes, an in-depth study with particular testing for each circumstance is required.

The restrictions for generating a total blood count are connected to the dataset's limitations. To begin, to perform a complete blood count, it would be necessary to have the ability to count and classify white cells. Its classification into monocytes, leukocytes, neutrophils, eosinophils, basophils, and lymphocytes, among others, is required for the exam to be complete. The dataset, however, does not give these classifications, instead of focusing on the contrasts between the three primary groups. Other volume-related numbers, such as MCV (mean corpuscular volume) and HCM (mean corpuscular hemoglobin), cannot be calculated due to a lack of data. This information can be derived from the data collection when using another dataset in future tasks.

## 5. Conclusions

This project attempted to use deep learning to assist health professionals by automating tasks so that they may focus on others. The blood count is one of the most important routine tests for detecting most illnesses. The best techniques to automate this activity were investigated in subsequent investigations. Deep learning algorithms were used to understand the blood count production process. All cells can be precisely enumerated by developing an intelligent computer model to recognize blood cells. This developed method enables decisions about a patient's health to be made. We can discover any imbalance in their levels by counting white, red, and platelets. More tests can be performed to validate these challenges if there is an aberrant component. Because of limitations in the dataset used and the general classification of white cells are not a comprehensive blood count, you can use these principles in future studies to collect new, more complex data or achieve another purpose. Another possibility is to use evaluation measures based on this technique, such as forecasts and true values. Based on this finding, the method utilized in this study can estimate the count in proportion to the volume and reproduce all of the information in a blood count.

## Figures and Tables

**Figure 1:** Perceptron.

**Figure 2:** Artificial neural network.

**Figure 3:** Convolutional neural network.

**Figure 4:** Interface of the prototype developed.

**Figure 5:** Defined parameters.

**Figure 6:** MSE and rMSE

**Figure 7:** Cell detection: WBC (a and b), RBC (c and d), and platelets (e and f).

## Data Availability

The data used to support the findings of this study are included within the article.
